# Problems and Measures of Traditional Culture Education and Mental Health Education in Colleges and Universities under the New Media Environment

This article has been retracted.

**DOI:** 10.1155/2022/3370481

**Published:** 2022-07-31

**Authors:** Xiang Zheng, Junxiao Bao, Jinli Wang

**Affiliations:** Chengde Medical University, ChengDe, Hebei 067000, China

## Abstract

The rapid development of information technology affects people's living habits. The new media based on information technology not only makes the traditional media suffer a serious impact but also breaks the constraints of traditional education methods. The orderly development of traditional culture education and mental health education activities in colleges and universities can play an important role in optimizing the ideological and cultural concepts and adjusting the psychological state of college students. It provides support and guarantees for college students to form scientific, cultural understanding concepts and good psychological quality. The gradual maturity of new media information transmission and distribution technology has profoundly influenced and changed the traditional cultural knowledge and mental health teaching work in colleges and universities, which has caused an extremely far-reaching real impact. This paper analyzes the problems of the traditional culture education and mental health education in colleges and universities under the new media environment. Then, the influence of new media on college students' traditional culture education and mental health education and its reasons are analyzed, and the corresponding countermeasures are put forward.

## 1. Introduction

Due to the continuous development of science and technology, the new media based on Internet information technology has become the most powerful media in the world like never before [1]. It brings a new communication mode and concept to the whole society. It is a media form that emerges under the support of a new technology system and has become the mainstream of media today [2]. Nowadays, people are accustomed to spending fragmented time learning knowledge and obtaining information. New media has become the primary choice for the public to understand the world. At present, under the background of the existing development and evolution of social and historical practices, the practical influence of traditional culture education in colleges and universities is coming to the fore [3].

Chinese culture has a long and profound history and is a valuable spiritual treasure for contemporary Chinese people [4]. The current education of Chinese traditional culture is difficult to combine with students' concrete learning life and concrete application due to its hollowness and abstraction. This makes students more resistant to the learning process [5]. In the context of globalization, western cultural ideas have more influence on college students' thoughts, which makes the development and inheritance of our traditional culture affected by the impact of western culture. College students are more active in the development of the Internet and are easily influenced by Western cultural ideas, and their behaviors and values are easily influenced by Western culture [6]. Therefore, through traditional culture education, students should firmly believe in the ideal of traditional culture and recognize and inherit our traditional culture.

Mental health education for college students in China is based on Western psychology as a theoretical foundation, and although it has achieved good educational results, the cultural ideas represented by Western psychology are not fully applicable to Chinese college students [7]. The development of social history originates from the process of human practice, and the culture formed in the creation of practice can shape a common personality that affects the individuals of the society through the forms of nation and state [8]. This shows that the common personality of the society has a subtle influence on each member of the society, which leads to a conscious adherence to the psychological characteristics of the personality of the society as a whole. Different cultural environments can form different psychological structures of personality, and people's psychological and behavioral characteristics are influenced by the cultural environment in which they live. Although culture itself is produced by human production and life activities, it also reacts to the development of human beings so that people of different countries, nationalities, and even regions have different thinking, psychology, and values [9]. Therefore, in mental health education, we should take the excellent traditional culture as the body and the western psychological theory as the use and form a mental health education system with our own characteristics.

Although it is difficult to study traditional culture education and mental health education in the new media environment, many scholars at home and abroad still explore it from different perspectives. Literature [10] holds that traditional culture can be used to enrich and improve the ideological education system. At the same time, traditional culture education can be integrated into the development and practice of new media by entering the classroom and integrating resources. Literature [11] argues that Internet culture has brought serious challenges to traditional culture and suggests creating databases of traditional cultural works, online classes, and e-commerce boosts to promote the transmission and development of traditional culture. Literature [12] suggests that the transmission of traditional culture on campus should be carried out by infiltrating culture into classroom teaching, organizing various cultural activities, and creating a good cultural environment on campus. Literature [13] studied the heritage of minority cultures and tea culture. Literature [14] showed that the psychological chat rooms set up in American colleges and universities can release the psychological stress of college students and effectively solve their psychological problems.

In today's fast-changing world, new media have promoted the innovation of college education and changed the ways and methods of traditional culture education. It is important to discuss the problems brought by new media to traditional culture education in colleges and universities and to propose effective countermeasures according to its causes. The traditional culture education in the new media environment is conducive to broadening the research perspective of education, exploring new carriers of education, and updating the means and methods of education. At the same time, the new media has made the cultural pattern in China more complicated, which has affected the development of mental health education for college students in China. At present, many of the psychological problems exposed by college students in China are closely related to the increasingly complex cultural environment. Therefore, it is an important task to carefully study the possible effects of its complexity on college students and to study the problems facing the development of college students' mental health education in a targeted manner.

This paper obtains first-hand information through a questionnaire survey to fully understand the actual situation of college students' use of new media. It analyzes the influence of new media on traditional culture education and mental health education in colleges and universities and the reasons for it, and puts forward effective methods to eliminate the problems in a targeted way.

This paper consists of five main parts: the first part is the introduction, the second part is state of the art, the third part is the methodology, the fourth part is result analysis and discussion, and the fifth part is the conclusion.

## 2. State of the Art

### 2.1. The Connotation, Extension, and Characteristics of New Media

New media is actually a relative concept, and being new is relative to the tradition and report, broadcast relative to a newspaper is a new media, television relative to broadcast is a new media, and network relative to television is a new media. In different time periods, there will always be a dominant media form [15]. New media is developing with the development of society. New media condense the new technological achievements created in the era and change the industrial structure in the society, directly affecting the way of information transmission in the era [16].

#### 2.1.1. The Connotation of New Media

New media refers to the current environment where media is prevalent and it covers all digital forms of media communication. In terms of its meaning, it not only has the advantages of traditional media but also has the characteristics of reciprocity and intermingling, flexibility and freedom, speed and efficiency, and has more open information, freer communication, richer communication methods, and more convenient communication speed compared to traditional media [17]. In general, new media is a concept proposed relative to traditional media. The current definition of new media is a media form that uses the network to disseminate information based on digital technology, Internet, and mobile Internet technology established under the development of global network technology, using digital mobile devices and other terminal carriers.

#### 2.1.2. Extent of New Media

The scope of new media is very large, and new media mainly includes fiber optic cable communication networks, graphic television, Internet, electronic computer communication networks, multimedia, and cell phone information interactive platforms, digital magazines and newspapers, digital movies, digital radio and television, microblogs, and Weibo [18].

#### 2.1.3. Characteristics of New Media

New media has the characteristics of a large amount of information, wide coverage, and massive information quantification. Its information dissemination has the advantages of extensiveness, convenience, and timeliness, as well as the flexibility of communication methods. For the public, it can be considered a media environment with strong topicality, novel content, and efficient communication. It mainly has the following characteristics.

*(1) Interactivity*. This is a distinctive feature of the new media, and effective information dissemination cannot be without interaction and communication between the two parties. In the previous media era, the communicator is the direct publisher of information, and the receiver of information is communicated, and the positioning between the two is very clear, with clear boundaries. This led to the problem that it was more difficult and less frequent for both parties to communicate, and the effect was weakened. In the new media environment, the boundaries between the two sides of communication are broken, and the interaction of information is synchronized so that the receiver can quickly spread the message after receiving it or spread it after modifying it according to his own understanding. And the two can also communicate with each other on topics of mutual concern using new media platforms such as Weibo and WeChat. This is conducive to the use and participation of users, and everyone can be the receiver and disseminator of information.

*(2) Openness*. New media make people's access to information more and more abundant, and express their opinions more and more convenient and free. The new media's information dissemination has broken the monopoly of traditional media on communication channels. In the past, there was a monopoly of information dissemination by certain groups and individuals, but now, this monopoly has been rapidly reduced. In the new media era, the way of communication is free and the content of the communication is open, but at the same time, the content is uneven, which increases people's selection and screening of good and bad information, and brings information burden to people.

*(3) Virtuality*. New media breaks the boundary between virtual and real world. In other words, new media technology also changes the way people interact with each other. In the new media environment, communication and interaction between people can be carried out in the virtual world, where everyone regularly hides their real situation and expresses it casually in the virtual world. In the virtual environment, it is good for people to express their ideas truly, for communicators to understand the dynamics of people's thoughts, and for the dissemination of positive information of interest to people from their needs so that the dissemination of information in the virtual world can better achieve meaningful results.

### 2.2. Challenges to the Dissemination of Traditional Culture Education

As a technology product, new media is a carrier and platform for communication, and the contents displayed on it are not objective and neutral. There are a lot of complicated content and information on new media, which will challenge universities to grasp the guidance of public opinion. In addition, the virtual nature of new media makes it possible for anyone to express his or her opinion freely, and many opinions and information will be spread rapidly, which brings challenges to the traditional education model [19].

#### 2.2.1. Challenges to Public Opinion Guidance

There are rich contents on the current new media, some of which are relatively healthy and positive, some of which are relatively negative and negative, and even some of which are used by western countries to promote the so-called freedom and equality ideas, which have posed challenges to the dissemination of ideology and the guidance of public opinion. Since college students themselves are busy with their studies in junior and senior high school, they do not have a deep understanding of society and their own three views are not fully formed, so they are easily influenced by the news on the new media platforms, and they are also easily confused by some bad thoughts that are well packaged in appearance, thus forming some bad ideologies and moral perceptions, or even the loss of ideal beliefs and faith [20]. In this context, traditional culture education in colleges and universities faces a great challenge in the dissemination of content, and whether the guidance of public opinion can be firmly grasped faces a test.

#### 2.2.2. The Virtualization of New Media Brings Challenges to the Education Model

New media is a platform for free speech, with openness and virtualization, on which everyone can express their ideas and opinions. These platforms seem to allow students to participate in discussions on various topics, but in reality, due to virtualization, some people express views that are not responsible and positive [21].

In the free space of the new media, students' right to speak is magnified, and many matters of immediate interest to students are closely followed and spread, and they have their own understanding and opinions on many hot topics, which makes it difficult for schools to adopt the traditional education model for indoctrination.

#### 2.2.3. The Plurality of New Media Communication Makes the Authority of Workers Challenged

In the traditional media communication of colleges and universities, we can see that there are heavy controls in the process of information collection, postproduction and editing, and publication, and each step has a gatekeeper for content review and presentation. The release of this information can be said to represent the official voice, which is relatively objective and rigorous, and the content of dissemination is generally positive and healthy. However, in the new media platform, although there are some monitoring means in China, it is unrealistic to carry out complete content control and audit due to the diversification and decentralization of communication subjects. Therefore, because there are too many subjects disseminating information, this can have an impact on students' acceptance, which leads to challenges to the authority of teachers' communication contents.

Traditional culture education can be controlled in the dissemination of information. Teachers disseminate educational information after repeated screening and deliberation before imparting it to students, which is a relatively single mode of communication with low interactivity, while current students often communicate through QQ, WeChat, and other platforms, and the communication process will be easily influenced by others, which brings challenges to teachers' information dissemination.

## 3. Methodology

### 3.1. Survey and Analysis of the Current Situation of Using New Media by College Students

#### 3.1.1. Basic Information of the Survey

The questionnaire survey through the questionnaire star app recovered 625 valid questionnaires, and the respondents include freshmen to seniors, 255 men and 370 women, including 148 freshmen, 161 sophomores, 159 juniors, and 157 seniors. The basic composition of the survey respondents is shown in Table 1.

#### 3.1.2. Analysis of Survey Results

*(1) The Popularity of New Media in College Student Groups*. To understand the popularity of new media, in the survey of “When you need to get information, what kind of media do you choose most of the time? The percentage of those who chose “new media” was 79.5%. The percentage of those who chose “traditional media” was 20.50% (Figure 1). This shows that new media has become an important medium for them to obtain information.

*(2) Time to Use New Media*. To understand the length of time new media is used, in the survey of “How many hours do you use new media every day?,” 15.68% chose “less than 2 hours,” 26.88% chose “2–4 hours,” 41.20% chose “4–6 hours,” and 16.24% chose “more than 6 hours.” The proportion of those who chose “more than 6 hours” was 16.24% (Figure 2). This shows that college students use new media for a long time every day and should plan their time reasonably.

*(3) Content Selection*. In order to understand the contents that college students often browse using new media, we surveyed “What do you usually browse when you use new media? (Multiple choice),” the survey results show that 78.87% of college students chose “leisure and entertainment.” The percentage of those who chose “official school information” was 71.21%. The proportion of those who chose “current news” was 58.42%, those who chose “social interaction” was 52.14%, and those who chose “other” was only 13.22% (Figure 3). The data analysis shows that college students pay more attention to leisure and entertainment and official school information when using new media, and college students have enriched their lives through new media platforms.

*(4) Impact on Values*. To understand the impact of new media on College Students' values, in the survey of “Do the different values you have been exposed to through new media have any influence on you?”, 42.11% of the respondents chose “not much influence,” and 28.56% chose “some influence.” 16.47% chose “a lot of influence,” and 12.86% chose “no influence.” Only 12.86% chose “no impact” (Figure 4). Through the analysis of the data, we can see that universities should actively guide college students to establish correct values.

*(5) Attitude Toward Information Confirmation Before Forwarding*. In order to understand college students' attitude towards confirming information before forwarding, in the survey of “Do you confirm the authenticity of information on new media platforms before forwarding or commenting?”, the percentage of those who chose “confirm” was 3.24%, “mostly confirm” was 30.78%, “mostly do not confirm” was 35.64%. The percentage of those who chose “not at all, it's all about their own preference” was 30.34% (Figure 5). From the above analysis, it can be seen that college students do not have a strong sense of discrimination when facing false information in new media.

*(6) Strengthen the Attitude of New Media Environment Regulation*. In order to fully understand college students' attitudes toward strengthening the regulation of the new media environment, in the survey of “Do you think there is a need to strengthen the regulation of the current new media environment?”, 41.22% of the respondents chose “more necessary,” 24.38% chose “very necessary,” 18.77% chose “generally necessary,” and 15.63% chose “nothing necessary” (Figure 6). Through the above analysis, it can be seen that the openness of new media makes the information dissemination out of control, and the widespread dissemination of bad information and negative social phenomena has brought certain troubles to college students. In order to ensure the “cleanliness” of the new media environment, continuous supervision is still needed.

*(7) Interaction*. In order to understand how college students use new media to participate in the interaction, in the survey of “Do you often like and retweet, comment and interact when browsing new media such as microblogs and Weibo?” The first one is “often” with 44.74%, followed by “occasionally” with 26.18%. The percentage of those who chose “hardly ever” was 17.25%, and the percentage of those who chose “never” was 11.83% (Figure 7). Through the above analysis, it can be seen that colleges and universities can use new media as a tool for communication between college students and educators so as to better understand students' voices and help them solve conflicts and difficulties in their lives. The negative remarks and negative thoughts of students can be guided to create a harmonious teacher-student relationship.

*(8) The Impact of New Media on College Students*. To understand the impact of the new media environment, when answering the question “What is the biggest impact of the new media on you? (Multiple choice),” 82.84% of the respondents chose “complicated information and impact on values,” ranking first. The percentage of those who chose “more interest in learning because of the richness of graphics” was 74.56%, the percentage of those who chose “more independent learning channels” was 61.20%, and the percentage of those who chose “easy to get addicted to new things and cut study time” was 53.44%. 53.44%, “facilitate communication and increase interaction between teachers and students” 39.75%, “affect physiological and psychological health” 26.36%, and “other” 7.22% (Figure 8). It can be seen that the negative information spread by the new media has brought a lot of trouble to college students. Gradually deviating from the mainstream values, serious problems such as a faith crisis may occur. The new media world is different from real life, and excessive indulgence in the virtual world wastes precious study time and distracts energy. There is no need to be responsible for what is said in the virtual social world and no need to be held accountable, and it is difficult to distinguish the truth from falsity in language, which tends to make college students lower their trust in others. At the same time, new media enriches the form of education, provides favorable conditions for college students' learning, increases acceptability and richness, and gives students a platform for independent learning.

*(9) The Impact of New Media on Traditional Culture Education*. In order to understand the impact of new media on traditional culture education, the question “What do you think are the problems in the use of new media in your school? (Multiple choice),” the top question was “Lack of novelty in content” with 72.11%, followed by “Lack of technology and staff on campus platform” with 55.82%. The percentage of those who chose “insufficient publicity” was 35.45%, 31.22% chose “not close to students' lives,” and 9.65% chose “other.” The percentage of those who chose “other” was 9.65% (Figure 9). This shows that the new media platforms do not really understand students' needs, and the format is rather rigid and cannot attract students' interest in learning.

### 3.2. Strive to Create a Fine Course of Traditional Culture

The questionnaire shows that 12.89% of college students are very willing to participate in the online courses and seminars related to Chinese excellent traditional culture sponsored by their schools, 48.77% of students will choose their favorite courses to participate in, and 32.23% of college students will occasionally participate in the course learning and discussion according to their own schedule (Figure 10), so as to achieve a deeper understanding of Chinese excellent traditional culture.

The analysis shows that a good popularization of traditional culture and education is very much in line with the demand. First, different media forms such as slides, animations, and campus cosplay shows can be used to promote the excellent Chinese traditional culture. Research shows that the new media mode with the network as the basic carrier can provide the most effective way of platform circulation. The difference in the effect of combining traditional culture and other cultural forms is becoming more and more obvious compared to the multiple media forms. In addition, the construction of a traditional cultural atmosphere can be achieved through the appreciation of classical masterpieces and the opening of book review activities or the organization of student groups to watch traditional culture-related film and television materials. Since the new media environment has the open concept feature, it can realize the effective undertaking of traditional knowledge by the college student group through the modernization and popularization of traditional knowledge.

### 3.3. Negative Effects of the New Media Environment on Mental Health Education

Although new media have brought a positive influence on the development and improvement of mental health education, mental health education needs to be cautious when combined with the new media background, and the diversity of new media in form and development has also brought negative influence to mental health education.

#### 3.3.1. College Students' Thinking and Behavior Are Impacted

On college campuses, it is the development, conflict, and integration of diversity that affects the thinking of college students. It manifests itself in the following ways.

First, there is a crisis of faith. The conflict of new media causes college students to be overwhelmed and unable to understand the conflict and contradiction between different cultural ideals and beliefs, and the cultural collision has greatly weakened college students' inherent sense of responsibility for their own lives. Second is the confusion of ethics and morality. In campus life, college students are unable to distinguish between good and bad things, focus only on their own interests and freedom, and ignore the sense of collective and social responsibility. Third, the moral evaluation criteria are blurred. The diversity of campus culture in colleges and universities causes the diversity of value choices of college students, which leads to the conflict of diverse cultures and values, which in turn leads to a series of chain reactions.

#### 3.3.2. The Value Conflict of University Campus Culture Shows a Tendency to Intensify

The spiritual power that campus culture brings to the university plays a vital role in the overall development of college students. With the continuous influx of various ideas and cultures, it promotes the exchange between different cultures and fills the types and contents of culture that are missing in contemporary campus culture. The influences and collisions of various cultures have opened up the horizons of university culture construction and thus changed the concept of campus culture, while at the same time, the conflict between values brought about by different cultures has intensified. The negative influences produced by various cultures in the exchange seriously hinder the fixation and formation of correct values of college students.

#### 3.3.3. The Influence of the Pluralism of Mass Media on Campus Culture

College students learn about society and themselves through various types of information provided by the mass media, thus expanding their own way of thinking. The mass media is a communication bridge that well combines school, students and society into one, making them inseparable and allowing students to fully integrate into society and realize their self-worth and social value. Therefore, despite the different identity backgrounds of students, all allow each individual to integrate their self-worth and social value organically. With the rapid development of mass media, there are some vulgar cultural contents in the society impacting the campus culture, which seriously affects students' judgment ability and makes college students lose their direction, thus leading to problems such as the pursuit of utilitarianism and hedonism. As a result, many students have problems in their thoughts and behaviors, not only indifferent to the interests of the country, the collective, and others but also develop extreme individualism in their own way, which leads to a wrong path of self-promotion.

## 4. Result Analysis and Discussion

### 4.1. Innovative Ways of Excellent Traditional Culture Education

For the education of excellent Chinese traditional culture, the rapid development of new media is both a great challenge and a new development opportunity to explore new ways of multidimensional development.

#### 4.1.1. Promoting Traditional Culture Education in New Media Territories

In the new media environment, websites, microblogs, WeChat, and various cultural APPs have broken the restrictions of time, place, and environment, and they are extremely fast, instant, diverse, and rich in content, making it easy to get information quickly.

In order to adapt to this excellent model, educators of Chinese traditional culture should keep in mind the “hard” original intention, “flexible” hand, and occupy new media positions from multiple angles, making it a new carrier and new channel for the public, especially young students to learn Chinese traditional culture. The new media will become a new vehicle and channel for the public, especially young students, to learn the excellent Chinese traditional culture.

#### 4.1.2. Innovative Forms of Education

Traditional didactic cultural education is prone to aesthetic fatigue and to a certain extent, stifles students' interest in learning. How to effectively transmit the excellent Chinese traditional culture to students, especially young students, so that they can really get into the ears, brains, and hearts, and identify with the excellent Chinese traditional culture from the heart, need to take advantage of the ever-changing new media technology.

*(1) Introduce Advanced Technology and Show the Value of Digitalization*. New media technology can digitize sound, pictures, text, and physical objects and use virtual reality technology and other high-tech means for cultural communication. With the help of three-dimensional animation and digital image technology, it can make audiences feel the cultural atmosphere in the real world and then identify with and love the excellent Chinese traditional culture.

*(2) Design Game App to Bring the Power of Digital Technology and Network into Play*. Online games are being integrated into the lives of the majority of young people, and games, as a carrier of cultural heritage, play no small role in spreading culture. China's 5,000 years of cultural history has created a treasure trove of inexhaustible cultural resources. Educators can design some game apps to bring Chinese traditional culture to the public. Through the games, players can experience the excellent Chinese traditional culture and make the traditional culture glow with attractiveness and vitality in playing.

*(3) Cultivate Cultural “Net Stars” and Release Network Energy*. In the new era, educators need to transform, and traditional culture educators should also become the new “Netflix” to communicate with young people and become responsible for bringing them closer to each other and transmitting mainstream values. For example, Professor Dai Jianye of Huazhong Normal University has been praised for his humorous and youthful approach to explaining the poems of Li Bai, Du Fu, and Tao Yuanming to his students. Therefore, more educators can learn from Professor Dai's approach and strive to interpret and promote the beautiful relevance of excellent Chinese traditional culture.

These cultural “net stars” show a unique way of expression and are loved by the public, more than anything else, because of the communication power of the Internet. New media integrates multiplatform and multitechnology, deeply integrating traditional culture and modern expressions, making traditional culture education transformed into cultural explosions and maximizing the effect of communication and education.

### 4.2. Traditional Culture into Mental Health Education Approach

#### 4.2.1. Create an Atmosphere for Learning Traditional Culture on Campus

The effective role of propaganda is becoming more and more prominent. The creation of an overall learning atmosphere on campus is conducive to making traditional culture deeply rooted in people's hearts and raising awareness and attention to traditional culture among teachers and students. Regularly update and push traditional culture-related knowledge, promote classic poems, character legends, fables, stories, and other excellent Chinese traditional culture, so that teachers and students in colleges and universities can be influenced by their eyes and ears, feel the same, accept traditional culture from deep inside consciously, and learn traditional culture actively.

#### 4.2.2. Increase the Efforts of Traditional Culture in the Classroom

Not only do primary and secondary schools need to offer compulsory courses on traditional culture, but universities also need to offer compulsory and elective courses that integrate the learning of traditional cultural knowledge in all courses. Traditional culture education can be linked to patriotic education and mental health education in university teaching, taking advantage of each other's strengths and highlighting the effects of specialized courses. The teaching design of mental health education class cannot be separated from the introduction of activities before the class, the inspiration of stories during the class, and a serious summary after the class, all of which can be properly introduced into traditional cultural knowledge, and the corresponding classic stories and legendary figures in traditional cultural knowledge can be integrated into it, which can not only learn traditional cultural knowledge but also improve the teaching quality and effect of mental health education class.

#### 4.2.3. Vigorously Carry Out Traditional Culture Practice Activities

The campus activities of colleges and universities are blossoming, and various clubs and associations are colorful and exciting, which can best attract the interest of college students and increase their active participation rate. Traditional culture-related clubs or associations are established in colleges and universities to attract students with special skills and interests and hold regular activities to promote traditional culture.

#### 4.2.4. Strengthen Students' Knowledge of Traditional Culture

Students are the ultimate beneficiaries and learners of traditional culture, and it is necessary to change students' learning attitudes and strengthen their knowledge of traditional culture. The excellent Chinese traditional culture condenses the wisdom of the ancients, is the essence and precipitation of ideas, and plays a role in promoting the healthy psychological growth of college students. As successors and builders of the socialist cause, college students must study and master traditional cultural knowledge in depth and internalize the knowledge into their own inherent cultivation, quality, and character. From the family, social, school, and personal levels, traditional culture is integrated into students' study and life, so that students can feel and experience the traditional culture Charm, improve students' interest in active learning, and infuse the essence of good traditional cultural knowledge into mental health education.

## 5. Conclusion

In the environment of rapid development of new media technology, it is important to take measures to improve the traditional cultural knowledge education of college students, to continuously improve and optimize the ideological and cognitive system of college students, and to support and guarantee the cultural knowledge literacy and mental health education of college students. To address the problems faced by traditional culture education and mental health education in the new media environment, this paper adopts the empirical research method, obtains first-hand information through a questionnaire survey, grasps the actual situation of college students' use of new media, analyzes the impact of new media on traditional culture education and mental health education of college students and its causes, and proposes operable methods and countermeasures to ensure that the research is based on evidence. Since new media are evolving with the progress of technology, the analysis of how to apply the advantages of new media to traditional culture education and mental health education in this paper is not comprehensive enough, which is also the focus of the next research work.

## Figures and Tables

**Figure 1:** Media type statistics.

**Figure 2:** New media usage time statistics.

**Figure 3:** Content selection of new media.

**Figure 4:** Influence of online information on values.

**Figure 5:** Attitude toward message confirmation before forwarding.

**Figure 6:** Attitudes towards better regulation of the new media environment.

**Figure 7:** Interactive survey results.

**Figure 8:** The impact of new media on college students.

**Figure 9:** Shortcomings of new media applications for traditional culture education.

**Figure 10:** Willingness to participate in online traditional culture course learning.

**Table 1:** Personnel structure of survey respondents.

Sample basic information		Number of people (625)	Percent (%)
Gender	Male	255	41
	Female	370	59

Grade	Freshman	148	23.68
	Sophomore	161	25.76
	Junior	159	25.44
	Senior	157	25.12

Subject type	Science and engineering	278	44.48
	Liberal arts	347	55.52

## Data Availability

The labeled data set used to support the findings of this study is available from the corresponding author upon request.
